The article "Exploring Pharmacological and Non-Pharmacological Approaches to Managing Hypertension During Pregnancy: A Systematic Review" was retracted in 2025. Reasons: unreliable results or conclusions; concerns about the authorship.

# Exploring Pharmacological and Non-Pharmacological Approaches to Managing Hypertension During Pregnancy: A Systematic Review

**DOI:** 10.7759/cureus.75534

**Published:** 2024-12-11

**Authors:** Saeeda Bano, Shahida Husain Tarar, Precious D Atung, Abdullah Shehryar, Abdur Rehman, Ahmad Irshad, Oluwatobiloba T Ogungbemi, Nahal Ijaz, Maryam Nour, Hafsah Abdirahiim Maalim

**Affiliations:** 1 Obstetrics and Gynecology, Sahiwal Medical College, Sahiwal, PAK; 2 Obstetrics and Gynecology, Aziz Bhatti Shaheed Teaching Hospital, Gujrat, PAK; 3 Obstetrics and Gynecology, Shenyang Medical College, Kaduna, NGA; 4 Internal Medicine, Allama Iqbal Medical College, Lahore, PAK; 5 Surgery, Mayo Hospital, Lahore, PAK; 6 General Surgery, Mayo Hospital, Lahore, PAK; 7 Internal Medicine, Caucasus International University, Tbilisi, GEO; 8 Medicine and Surgery, Avicenna Hospital, Lahore, PAK; 9 Family Medicine, Emergency Medicine, Internal Medicine, Psychiatry, John F. Kennedy University School of Medicine, Williemstad, CUW; 10 Emergency Medicine, Henry Ford Health System, Detroit, USA; 11 Internal Medicine, Omdurman Islamic University, Khartoum, SDN

**Keywords:** dash diet, labetalol, preeclampsia, pregnancy hypertension, remote monitoring

## Abstract

This systematic review aimed to explore the efficacy of both pharmacological and non-pharmacological interventions in managing hypertension during pregnancy. It analyzed high-quality randomized controlled trials (RCTs), focusing on outcomes related to maternal and fetal health. The findings demonstrated that antihypertensive medications, particularly labetalol and nifedipine, effectively reduced the risks of severe preeclampsia (PE), preterm birth, and other complications. Remote monitoring of blood pressure (BP) showed promise in improving postpartum care and addressing health disparities. While dietary interventions such as the Dietary Approaches to Stop Hypertension (DASH) diet offered metabolic benefits, their impact on preventing PE was inconclusive. The review highlights the need for a comprehensive approach to hypertension management, integrating medication, lifestyle interventions, and innovative monitoring strategies. It also emphasizes the importance of further research to refine non-pharmacological interventions and assess their long-term effectiveness. We believe these insights will help guide clinical practice, enhance maternal and fetal outcomes, and inform future research directions.

## Introduction and background

Hypertension during pregnancy is a significant clinical concern, affecting approximately 5-10% of all pregnancies and representing a leading cause of maternal and fetal morbidity and mortality worldwide [1]. The condition encompasses chronic hypertension, gestational hypertension, and preeclampsia (PE), with each presenting unique challenges to maternal and fetal health. Uncontrolled hypertension during pregnancy is associated with adverse outcomes such as preterm birth, placental abruption, intrauterine growth restriction, and an increased risk of cardiovascular diseases in later life [2].

Traditionally, pharmacological interventions have formed the cornerstone of hypertension management, with antihypertensive agents like labetalol, methyldopa, and nifedipine being commonly prescribed [3]. However, the potential risks of medication exposure during pregnancy necessitate exploring alternative or complementary non-pharmacological strategies. Lifestyle modifications, dietary interventions such as the Dietary Approaches to Stop Hypertension (DASH) diet and Mediterranean diet, and remote blood pressure (BP) monitoring have shown promise as non-pharmacological approaches in managing pregnancy-related hypertension [4].

Despite significant advances in research and clinical guidelines, there remains considerable variability in the application and effectiveness of these strategies across different settings and patient populations. Therefore, a comprehensive evaluation of both pharmacological and non-pharmacological approaches is crucial for optimizing maternal and fetal outcomes [5]. Hence, this systematic review aims to synthesize evidence from recent randomized controlled trials (RCTs) to provide a clearer understanding of the effectiveness of these interventions while identifying potential gaps and areas for future research.

This review adopted a Population, Intervention, Comparison, and Outcome (PICO) framework [6]. The Population (P) includes pregnant women diagnosed with any form of hypertension, such as chronic hypertension, gestational hypertension, or PE. The Interventions (I) encompass both pharmacological and non-pharmacological approaches. Pharmacological interventions include commonly prescribed antihypertensive agents like labetalol, nifedipine, methyldopa, hydralazine, and clonidine. Non-pharmacological strategies comprise lifestyle interventions, dietary modifications such as the DASH and Mediterranean diets, and technological solutions like remote monitoring. Comparison (C) involves standard care or alternative management approaches, including other pharmacological agents or standard in-office surveillance in the case of non-pharmacological interventions. The primary Outcomes (O) include BP control, the incidence of severe hypertension, PE, and maternal and fetal outcomes like preterm birth and intrauterine growth restriction. Secondary outcomes include maternal quality of life, adherence to interventions, and long-term cardiovascular health, providing a comprehensive understanding of the impact of these management strategies.

The primary objective of this systematic review is to evaluate the roles and comparative effectiveness of pharmacological and non-pharmacological interventions in managing hypertension during pregnancy. Specifically, the review aims to assess the impact of antihypertensive agents on maternal and fetal outcomes, with a particular focus on their safety, efficacy, and optimal timing of initiation. The review also seeks to examine the efficacy of non-pharmacological strategies, such as dietary interventions, lifestyle modifications, and remote monitoring, in achieving BP control and reducing adverse pregnancy outcomes. By synthesizing the existing evidence, this review intends to identify gaps in current research and highlight areas requiring further investigation to inform clinical practice. Ultimately, the goal is to provide clinicians and researchers with evidence-based insights to improve maternal and fetal outcomes and guide the development of comprehensive, tailored management strategies for hypertension in pregnancy.

## Review

Materials and methods

Search Strategy

The search strategy for this systematic review was designed to comprehensively identify relevant RCTs and clinical studies evaluating the roles of pharmacological and non-pharmacological interventions in the management of hypertension during pregnancy. A systematic search was conducted across major electronic databases, including PubMed, MEDLINE, Cochrane Central Register of Controlled Trials (CENTRAL), Embase, and Scopus.

The search terms combined MeSH terms and free-text keywords related to pregnancy hypertension, such as “chronic hypertension in pregnancy,” “gestational hypertension,” “preeclampsia,” “hypertensive disorders of pregnancy,” as well as specific intervention terms like “antihypertensive therapy,” “labetalol,” “nifedipine,” “methyldopa,” “clonidine,” “hydralazine,” and non-pharmacological strategies including “DASH diet,” “Mediterranean diet,” “lifestyle interventions,” and “remote monitoring.” Boolean operators (AND, OR) were employed to combine search terms effectively, and the search was limited to studies published in English over the last 10 years to ensure the inclusion of recent evidence. Reference lists of relevant articles and systematic reviews were manually screened to capture additional eligible studies. The Preferred Reporting Items for Systematic Reviews and Meta-Analyses (PRISMA) guidelines were followed to ensure a robust and transparent search process, aiming to minimize bias and maximize the retrieval of pertinent studies for review [7].

Eligibility Criteria

The eligibility criteria for this systematic review were established to include studies focusing on the management of hypertension in pregnant women using pharmacological and non-pharmacological interventions. We included RCTs and clinical trials published in English involving pregnant women diagnosed with any form of hypertension, including chronic hypertension, gestational hypertension, and PE. Eligible studies had to assess the effectiveness, safety, and maternal-fetal outcomes associated with antihypertensive medications such as labetalol, nifedipine, methyldopa, hydralazine, and clonidine. Additionally, studies evaluating non-pharmacological strategies like the DASH diet, Mediterranean diet, lifestyle modifications, and remote BP monitoring were considered. We focused on studies reporting primary outcomes such as BP control, incidence of PE, severe hypertension, preterm birth, and maternal-fetal complications. Secondary outcomes included adherence to interventions, maternal quality of life, and long-term cardiovascular health.

Exclusion criteria included studies involving women with pre-existing cardiovascular or renal conditions unrelated to pregnancy, case reports, observational studies, editorials, and articles published in languages other than English. Studies involving interventions that did not focus primarily on BP control or maternal-fetal outcomes were excluded. Additionally, reviews, meta-analyses, and studies conducted before 2010 were not considered, as the aim was to incorporate the most recent and relevant evidence. Studies lacking clear outcome measures or data on key variables related to hypertension and pregnancy management were excluded to maintain the integrity and specificity of the review. This selection process ensured a focus on high-quality, clinically relevant evidence to address the research question comprehensively.

Data Extraction

Data extraction was carried out using a standardized extraction form to capture all pertinent information from each selected study. Two independent reviewers extracted data, focusing on study characteristics such as author details, year of publication, study design, sample size, and population characteristics, including type and severity of hypertension in pregnancy. Detailed information on interventions, including specific pharmacological agents (labetalol, nifedipine, methyldopa, hydralazine, clonidine) and non-pharmacological strategies (DASH diet, Mediterranean diet, lifestyle modifications, remote monitoring), was meticulously recorded. Comparison groups, if applicable, were noted along with control or alternative interventions. Primary outcomes included BP control, incidence of severe hypertension, PE, and maternal-fetal complications, while secondary outcomes comprised adherence rates, maternal quality of life, and long-term cardiovascular health. For each study, key findings relevant to the efficacy, safety, and impact of interventions were summarized, ensuring consistency and accuracy in the extraction process. Any discrepancies between reviewers were resolved via discussion or consultation with a third reviewer to maintain the rigor and reliability of the extracted data.

Data Analysis and Synthesis

Data analysis and synthesis for this systematic review were conducted using a narrative synthesis approach given the diversity in interventions and outcome measures across the included studies. The primary step involved categorizing studies based on the type of intervention - pharmacological or non-pharmacological - and then organizing them according to specific treatments, such as antihypertensive medications or lifestyle modifications. For each category, the effectiveness of interventions was evaluated by comparing the reported primary outcomes, including BP control, reduction in severe hypertension, incidence of PE, and maternal-fetal outcomes.

Secondary outcomes, such as maternal quality of life, adherence to interventions, and long-term cardiovascular health, were assessed qualitatively to identify trends, patterns, and variations. Key findings were synthesized by highlighting the comparative effectiveness, safety profiles, and impact of different management strategies. Any inconsistencies or significant heterogeneity between studies were explored to understand their potential causes, such as differences in study design, population characteristics, or intervention protocols. The synthesized data were then used to draw conclusions about the relative benefits of various interventions and to identify gaps in the current evidence, guiding recommendations for future research and clinical practice.

Results

Study Selection Process

The search initially elicited 419 records from various databases, including PubMed, MEDLINE, CENTRAL, Embase, and Scopus (Figure 1). After removing 70 duplicate records, 349 were screened, and 88 were excluded. Of the 261 reports sought for retrieval, 103 were not retrieved. From the remaining 158 reports, several studies were excluded due to the following reasons: pre-existing conditions unrelated to pregnancy, non-English articles, irrelevant study types, interventions not focused on BP control, reviews or pre-2010 studies, and lack of clear outcome measures. Ultimately, 10 new studies were included in the final analysis.

**Figure 1:** The PRISMA flow diagram depicting the study selection process PRISMA: Preferred Reporting Items for Systematic Reviews and Meta-Analyses

Characteristics of the Selected Studies

The selected studies included a range of multicenter RCTs and secondary analyses, focusing on pregnant and postpartum women with various forms of hypertension: chronic hypertension, gestational hypertension, and PE. These studies examined the effectiveness of different pharmacological treatments such as labetalol, nifedipine, methyldopa, clonidine, and hydralazine, as well as non-pharmacological interventions including lifestyle modifications, dietary approaches like the DASH diet, and remote monitoring of BP. The primary outcomes of interest across studies included BP control, incidence of severe PE, preterm birth, and fetal or neonatal complications. Secondary outcomes explored various maternal and neonatal health indicators such as lipid profiles, glycated hemoglobin levels, and adherence to interventions. Key findings emphasized the comparative effectiveness of the interventions, the role of self-monitoring in achieving long-term BP control, and the need for personalized approaches in low-resource settings (Table 1).

**Table 1:** Summary of the included studies BP: blood pressure; CHAP: Chronic Hypertension and Pregnancy; CRP: C-reactive protein; DASH: Dietary Approaches to Stop Hypertension; DBP: diastolic blood pressure; GH: glycated hemoglobin; GP: glutathione peroxidase; ICU: intensive care unit; MAP: mean arterial pressure; PDM: pre-existing diabetes mellitus; PE: preeclampsia; PRISMA: Preferred Reporting Items for Systematic Reviews and Meta-Analyses; RCT: randomized controlled trial; RoB 2: Cochrane Risk of Bias 2 tool; SBP: systolic blood pressure

Authors	Study design	Population	Intervention	Comparison	Primary outcomes	Secondary outcomes	Key findings
Sanusi et al., 2024 [8]	Multicenter RCT	Pregnant women with mild chronic hypertension (BP: <160/105 mmHg)	Antihypertensive treatment (primarily labetalol or nifedipine) to achieve a BP goal of <140/90 mmHg	No treatment unless BP reached severe levels	Composite risk of severe PE, preterm birth <35 weeks, placental abruption, and fetal/neonatal death	None specifically stated	Antihypertensive treatment to achieve BP <140/90 mmHg significantly reduced the risk of severe PE, indicated preterm birth, placental abruption, and fetal/neonatal death compared to no treatment unless BP became severe. Recommended by US professional societies
Easterling et al., 2019 [9]	Multicenter, parallel-group, open-label RCT	Pregnant women (≥18 years, ≥28 weeks gestation) with severe hypertension (SBP ≥160 mmHg or DBP ≥110 mmHg)	Oral antihypertensives: nifedipine (10 mg hourly), labetalol (200 mg hourly), or methyldopa (1000 mg single dose)	Comparison between the three oral drugs	BP control (120-150 mmHg systolic and 70-100 mmHg diastolic) within 6 hours without adverse events	Occurrence of serious adverse events, such as intrapartum seizures and stillbirths	Nifedipine achieved the primary outcome more frequently than methyldopa. No significant difference in primary outcomes between nifedipine and labetalol, or labetalol and methyldopa. All three oral drugs were viable options in low-resource settings
Donel et al., 2023 [10]	Multicenter, double-blind RCT	Pregnant women with severe PE in hypertensive emergencies	Nifedipine (3 doses), labetalol (3 doses), or hydralazine (3 doses) administered within one hour at 20-minute intervals	Comparison between the three drugs for BP reduction effectiveness	Reduction in MAP by 20%	Failure to achieve 20% MAP reduction after third dose; incidence of adverse events	Nifedipine was most effective for single-dose BP reduction, while hydralazine was most effective when administered in triple doses. Each drug reduced BP significantly, but effectiveness varied based on dosing strategy
Arkerson et al., 2023 [11]	Multisite RCT	Postpartum patients with hypertensive disorders of pregnancy	Remote monitoring of BP using a web-enabled smartphone platform	In-office BP assessment	Rate of BP ascertainment within 10 days of postpartum discharge	Rates of antihypertensive medication initiation, readmission, and additional visits for hypertension	Remote monitoring increased postpartum BP ascertainment rates compared to in-office checks (91.7% vs. 58.4%). No significant differences in readmission rates or medication initiation. Promoted health equity, eliminating racial disparities seen with in-office monitoring
Belfort et al., 2023 [12]	Randomized, controlled, single-blind trial	Pregnant women with PDM	DASH diet with higher fiber, unsaturated fats, calcium, magnesium, and potassium	Standard diet with similar macronutrient distribution (45-65% carbohydrates, 15-20% protein, 25-30% lipids)	Incidence of PE	BP, GH, serum lipids, GP, and CRP	The DASH diet showed a trend toward reducing PE incidence (though not statistically significant). GP levels increased significantly, indicating potential metabolic benefits, while GH levels decreased similarly in both groups. No difference in PE incidence was observed between groups
Dodd et al., 2014 [13]	Multicenter RCT	Overweight or obese pregnant women (BMI: ≥25), 10+0 to 20+0 weeks' gestation	Comprehensive antenatal dietary and lifestyle intervention delivered by research staff	Standard care according to local guidelines without lifestyle information	Incidence of infants born large for gestational age (birth weight ≥90th percentile)	Birth weight >4000 g, hypertension, PE, gestational diabetes	The lifestyle intervention did not significantly reduce the risk of delivering a large-for-gestational-age infant but reduced the likelihood of infants weighing above 4000 g. No significant differences in maternal pregnancy and birth outcomes were observed
Kitt et al., 2023 [14]	Randomized, open-label, blinded end-point trial	Postpartum women with a history of PE or gestational hypertension requiring antihypertensive medication	Self-monitoring with physician-optimized antihypertensive titration	Usual postnatal care	24-hour mean DBP at 9 months postpartum	24-hour mean SBP	The intervention group had significantly lower diastolic (-5.8 mmHg) and systolic (-6.5 mmHg) BP compared to usual care. Self-monitoring with physician-guided adjustments resulted in better long-term BP control
Noronha Neto et al., 2017 [15]	Triple-blind RCT	Postpartum women with hypertensive disorders of pregnancy and severe hypertension (SBP ≥180 mmHg or DBP ≥110 mmHg)	Clonidine	Captopril	Frequency of very high BP episodes during obstetric ICU stay	Reduction in SBP, need for sodium nitroprusside, adverse reactions	Clonidine showed a non-significant reduction in high BP episodes compared to captopril, with a significantly lower SBP on the third postpartum day. Both clonidine and captopril were safe and effective for severe postpartum hypertension management
Pels et al., 2018 [16]	Secondary analysis of the CHIPS RCT data	Pregnant women with nonsevere chronic or gestational hypertension	Less-tight control (target DBP of 100 mmHg)	Tight control (target DBP of 85 mmHg)	Major maternal and perinatal outcomes based on timing of antihypertensive initiation	Birth weight <10th percentile, preterm birth, perinatal death, and high-level neonatal care >48 hours	Delaying antihypertensive therapy until later in pregnancy showed fewer low birth weight babies but an increased risk of preterm birth with less tight control. No gestational age was identified at which less tight control was preferred for optimizing maternal or perinatal outcomes
Wang et al., 2018 [17]	RCT with a cohort analysis	Pregnant women with gestational hypertension, mild PE, or severe PE	Oral nifedipine vs. intravenous labetalol	Comparison of the two antihypertensive therapies for severe PE	BP reduction to target levels, maternal and neonatal outcomes	Lipid profile and cytokine levels linked to severity of hypertensive disorders	Both oral nifedipine and intravenous labetalol were effective and safe in reducing BP in severe PE. The study suggests a potential role of lipid profiles and cytokines in assessing the severity of hypertensive disorders. Nifedipine use warrants further study

Discussion

Our findings highlight the comparative effectiveness of various pharmacological and non-pharmacological interventions in managing hypertension during pregnancy. Antihypertensive treatments, such as labetalol (Normodyne®, 100-400 mg twice daily) and nifedipine (Procardia XL®, 10-30 mg twice daily), demonstrated significant reductions in the risk of severe PE, preterm birth, placental abruption, and fetal/neonatal death in women with mild chronic hypertension, as elaborated by Sanusi et al. [8]. Similarly, in cases of severe hypertension, oral nifedipine was effective in achieving BP control, with results comparable to labetalol and methyldopa, as demonstrated in a low-resource setting study by Easterling et al. [9]. While they did not establish the superiority of nifedipine over labetalol or methyldopa, the ease of administration and rapid onset of action make nifedipine a practical option in emergencies. For hypertensive emergencies in severe PE, nifedipine (10 mg hourly) showed the greatest efficacy for single-dose reductions in BP, while hydralazine (Apresoline®, 5-10 mg intravenously every 20-30 minutes) was most effective when administered in multiple doses, as reported by Donel et al. [10].

It is essential to consider the potential teratogenicity and fetotoxicity of these drugs. Although labetalol and methyldopa are considered safe during pregnancy, nifedipine and hydralazine may occasionally cause adverse effects such as maternal hypotension, fetal distress due to sudden BP changes, and placental hypoperfusion. Methyldopa has been associated with fatigue and depression in some patients, while hydralazine is linked to reflex tachycardia and fluid retention. This underscores the importance of individualized treatment and careful monitoring during therapy to minimize risks and optimize maternal-fetal outcomes.

Non-pharmacological strategies like remote monitoring enhanced postpartum BP ascertainment and promoted health equity, eliminating racial disparities compared to in-office monitoring as shown by Arkerson et al. [11]. Although dietary interventions like the DASH diet and antenatal lifestyle advice did not significantly reduce PE incidence or adverse maternal outcomes, they showed trends toward metabolic benefits and lower rates of large-for-gestational-age infants, as revealed by Belfort et al. [12] and Dodd et al. [13]. Moreover, Kitt et al. [14] showed that self-monitoring with physician-guided antihypertensive adjustments achieved better long-term BP control in postpartum women. Collectively, these findings underscore the benefits of a tailored approach that integrates both pharmacological and non-pharmacological interventions to optimize maternal and fetal outcomes in managing hypertension during pregnancy.

This review's findings align closely with existing literature that underscores the importance of individualized management of hypertension in pregnancy using both pharmacological and non-pharmacological strategies [1]. Current guidelines, such as those from the American College of Obstetricians and Gynecologists (ACOG), recommend antihypertensive treatment for chronic hypertension during pregnancy to achieve BP targets below 140/90 mmHg [18], which is consistent with the significant risk reduction seen in the Chronic Hypertension and Pregnancy (CHAP) trial by Sanusi et al. (2024). Similarly, the preference for oral nifedipine and labetalol for severe hypertension in pregnancy corroborates previous recommendations favoring these medications due to their safety profiles and effectiveness in BP control [19,20].

However, the review also highlighted differences in the effectiveness of antihypertensive agents depending on dosage strategies and resource settings, echoing the findings of earlier studies suggesting the need for tailored treatment approaches. Notably, this review endorses the growing evidence for remote monitoring as an effective method to enhance postpartum BP management and promote health equity, findings that resonate with studies advocating the use of digital health interventions [21]. Conversely, while dietary interventions like the DASH and Mediterranean diets showed trends toward metabolic benefits, the lack of statistically significant reductions in PE incidence diverges from some smaller studies reporting greater effectiveness [22]. These variations indicate the complexity of non-pharmacological interventions and the influence of study designs, populations, and adherence levels on outcomes, emphasizing the need for further high-quality research to refine these strategies.

The findings from this review have important implications for clinical practice, particularly in refining hypertension management strategies during pregnancy. The demonstrated effectiveness of antihypertensive treatments like labetalol and nifedipine in reducing severe PE and adverse fetal outcomes supports current guidelines that recommend targeting BP below 140/90 mmHg. However, these treatments are not without potential risks. For mothers, antihypertensive medications can lead to side effects such as fatigue, dizziness, and in rare cases, hypotension or reflex tachycardia, which may require careful dose adjustments. For the fetus, there is a potential risk of impaired placental perfusion with aggressive BP lowering, which could lead to intrauterine growth restriction or preterm birth in some cases. Additionally, the efficacy of remote monitoring in enhancing postpartum BP control suggests integrating digital health tools into routine care, which could improve accessibility and health equity [23].

Non-pharmacological interventions, such as dietary modifications and lifestyle counseling, offer additional benefits but also present potential challenges. While dietary interventions like the DASH diet are generally safe, poor adherence or inadequate nutritional adjustments could result in suboptimal BP control, indirectly affecting both maternal and fetal health. Similarly, lifestyle modifications may be difficult to implement consistently due to socioeconomic barriers or lack of access to resources. Overall, these findings reinforce the importance of a multifaceted approach to hypertension management, combining pharmacological treatments with supportive interventions while considering the potential adverse effects on both the mother and baby. Such strategies aim to improve maternal and fetal health outcomes while minimizing risks [24].

This systematic review demonstrates several key strengths, including the use of a robust and comprehensive methodology adhering to PRISMA guidelines, which ensured a structured and transparent approach to study selection and data synthesis. By focusing exclusively on high-quality RCTs, the review aimed to provide strong evidence for clinical decision-making. Additionally, the use of the Cochrane Risk of Bias 2 (RoB 2) tool enabled a rigorous assessment of study quality, minimizing the impact of methodological biases on the overall findings [25]. However, there are limitations to consider, such as the variability in study designs, sample sizes, and the diversity of interventions included, which may introduce heterogeneity in the results. Furthermore, the open-label nature of some trials and differences in reporting outcomes could contribute to biases. These limitations, combined with the lack of meta-analyses, may affect the generalizability and comparability of the findings. Future research should focus on more standardized outcome measures and explore additional interventions to enhance the consistency and applicability of evidence in clinical practice.

Future research should prioritize well-designed RCTs with larger sample sizes and longer follow-up periods to better assess the long-term effects of various interventions for managing hypertension during pregnancy. Studies should explore the integration of both pharmacological and non-pharmacological approaches, such as combining antihypertensive medication with remote monitoring or dietary interventions, to identify synergistic effects that could improve maternal and fetal outcomes. Research focusing on diverse clinical settings and populations is key to evaluating the generalizability of interventions, particularly in low-resource environments where access to certain medications and technologies may be limited [26]. Additionally, standardizing outcome measures and adopting patient-centered endpoints, such as quality of life and maternal satisfaction, would provide a more holistic understanding of treatment effectiveness. Addressing these gaps will help refine clinical guidelines and advance personalized, evidence-based care for pregnant women with hypertension.

## Conclusions

This review underscores the importance of a multifaceted approach to managing hypertension during pregnancy, integrating both pharmacological and non-pharmacological interventions to optimize maternal and fetal outcomes. The findings affirm the efficacy of antihypertensive medications such as labetalol (oral, 100-400 mg twice daily) and nifedipine (10-30 mg twice daily) in reducing the risk of severe complications, including PE, preterm birth, and placental abruption. For hypertensive emergencies, intravenous hydralazine (5-10 mg every 20-30 minutes) and intravenous labetalol (20 mg initially, followed by incremental doses of 40 mg and 80 mg every 10 minutes) are commonly employed to achieve rapid BP control. The potential of remote monitoring to enhance postpartum care and promote health equity is also significant, highlighting its role as a complementary strategy in hypertension management. However, while dietary and lifestyle interventions show promising metabolic benefits, their impact on key maternal and fetal outcomes remains uncertain and needs further research. Overall, this review provides valuable insights that can inform clinical practice, encouraging tailored and evidence-based strategies to improve the management of hypertension in pregnancy, ultimately aiming to enhance patient safety and healthcare outcomes.
